The article "Human immunodeficiency virus-positive secondary syphilis mimicking cutaneous T-cell lymphoma" was published in 2015. Journal: Diagn Pathol.

# Human immunodeficiency virus-positive secondary syphilis mimicking cutaneous T-cell lymphoma

**DOI:** 10.1186/s13000-015-0419-5

**Published:** 2015-10-08

**Authors:** Michiko Yamashita, Yoshiyuki Fujii, Keiji Ozaki, Yoshio Urano, Masami Iwasa, Shingen Nakamura, Shiro Fujii, Masahiro Abe, Yasuharu Sato, Tadashi Yoshino

**Affiliations:** Division of Diagnostic Pathology, Tokushima Red Cross Hospital, 103, Irinokuchi, Komatsushima-cho, Komatsushima-shi, Tokushima, 7738502 Japan; Division of Hematology, Tokushima Red Cross Hospital, Tokushima, Japan; Division of Dermatology, Tokushima Red Cross Hospital, Tokushima, Japan; Division of Hematology, Tokushima University Hospital, Tokushima, Japan; Department of Pathology, Okayama University Graduate School of Medicine, Dentistry, and Pharmaceutical Sciences, Okayama, Japan

**Keywords:** Human immunodeficiency virus (HIV), HIV-1, Syphilis, Co-infection, Skin lesions, CD8, Malignant secondary syphilis, Lues maligna, Cutaneous T-cell lymphoma

## Abstract

Malignant syphilis or lues maligna is a severe form of secondary syphilis that was commonly reported in the pre-antibiotic era, and has now reemerged with the advent of the human immunodeficiency virus (HIV) epidemic. However, the characteristic histopathological findings of malignant syphilis remain controversial. The aim of this case report was to clarify the clinical and histopathological findings of HIV-positive malignant secondary syphilis. A Japanese man in his forties complained of fever, skin lesions, headache, and myalgia without lymphadenopathy during the previous 4 weeks. The skin lesions manifested as erythematous, nonhealing, ulcerated papules scattered on his trunk, extremities, palm, and face. Although the skin lesions were suspected to be cutaneous T-cell lymphomas on histological analyses, they lacked T-cell receptor Jγ rearrangement; moreover, immunohistochemical analyses confirmed the presence of spirochetes. The patient was administered antibiotics and anti-retroviral therapy, which dramatically improved the symptoms. On the basis of these observations of the skin lesions, we finally diagnosed the patient with HIV-associated secondary syphilis that mimicked cutaneous T-cell lymphoma. The patient’s systemic CD4+ lymphocyte count was very low, and the infiltrate was almost exclusively composed of CD8+ atypical lymphocytes; therefore, the condition was easily misdiagnosed as cutaneous lymphoma. Although the abundance of plasma cells is a good indicator of malignant syphilis on skin histological analyses, in some cases, the plasma cell count may be very low. Therefore, a diagnosis of malignant secondary syphilis should be considered before making a diagnosis of primary cutaneous peripheral T-cell lymphoma or lymphoma associated with HIV infection.

The article "Human immunodeficiency virus-positive secondary syphilis mimicking cutaneous T-cell lymphoma" was published in 2015. Journal: Diagn Pathol.

## Background

Lues maligna, also known as malignant secondary syphilis or ulceronodular syphilis, is an aggressive and lethal form of secondary syphilis. Although it was previously eradicated in developed countries with the introduction of antibiotics, it has reemerged recently [1–3]. The disease manifests as multiple skin lesions on the face and extremities following a short incubation period; these lesions are characterized by a nonhealing central ulcer with peripheral extension and a thick, crusty covering. The palms and soles are often affected, and fever, myalgia, and headache commonly occur. Compatible gross and microscopic morphology, a high antibody titer on serologic tests for syphilis, Jarisch-Herxheimer reaction following treatment, and dramatic response to antibiotic therapy are classical criteria used for diagnosing malignant secondary syphilis [1, 3].

Since the 1900s, co-infection with malignant secondary syphilis and human immunodeficiency virus (HIV) has been more frequently reported; with HIV infection and lues maligna, the outcomes are even poorer than previously reported with lues maligna alone in the pre-HIV period [4]. There has been a recent increase in the number of syphilis and HIV co-infection cases, and estimates indicate that 16 % of all patients with syphilis and 28 % of male patients with syphilis in the United States are HIV positive [5]. In a Japanese clinical study conducted from 1986 to 2000, 40.3 % of HIV-1-positive patients also tested positive for rapid plasma reagin (RPR) [6]. The combination of syphilis and HIV is particularly dangerous because eroded secondary syphilids increase the risk of HIV infection, and HIV can alter the natural history of syphilis [7]. A new syphilis infection increases the viral load of HIV and decreases CD4+ cell counts in HIV-infected patients [8]. Potentially because of B-cell dysregulation, the RPR test tends to be masked by the prozone phenomenon, especially in patients with HIV [9]. Malignant secondary syphilis and central nervous system syphilis are both lethal conditions. Therefore, it has been suggested that all HIV-positive syphilis patients should be treated with a penicillin-based regimen that is adequate for the treatment for neurosyphilis [10].

Skin lesions mimicking lymphoma have been reported in a *simple* infection of either syphilis or HIV. The *simple* syphilis, particularly in secondary syphilis, induces generalized lymphadenopathy, and lymphocyte-dominant skin infiltration admixed with neutrophils, histiocytes, and plasma cells, which can easily be interpreted as lymphoma cutis by pathologists [11]. The abundance of neutrophils seen in these malignant syphilis cases was also observed in the present case [11, 12]. In contrast, lymphoid proliferative lesions in a *simple* HIV infection that are characterized by polyclonal CD8+ lymphocytes that improve with only antiretroviral therapy (ART) have also been reported and called lymphomas associated with HIV infection, diffuse infiltrative lymphocytosis syndrome, and CD8+ pseudolymphoma [13].

The article "Human immunodeficiency virus-positive secondary syphilis mimicking cutaneous T-cell lymphoma" was published in 2015. Journal: Diagn Pathol.

In syphilis and HIV *co*-*infection*, skin lesions have been reported as atypical cutaneous lymphoproliferative disorders in patients with HIV [14]. Tosca et al. reported that lymphocytes can be of both the CD4 and CD8 types, [15] whereas Muche et al. reported that 85 % of the skin-infiltrating lymphocytes in HIV patients were CD8+ T-cells [16]. However, the histopathological findings remain controversial. Recently, we encountered a case of HIV-positive malignant secondary syphilis that histologically mimicked cutaneous peripheral T-cell lymphoma. Here, we report the clinical and pathological manifestation of the case and describe the correlation with the 4^th^ edition of the World Health Organization (WHO) tumor classification [17].

## Case presentation

### Clinical summary

A married Japanese man in his forties presented with fever and 1- to 5-cm, well-demarcated, round-to-oval erythematous pruritic skin macules on his trunk and upper extremities (Fig. 1a). He complained of severe headache and arthralgia and reported low-grade fever, fatigue, and weight loss during the previous 4 weeks. Superficial lymphadenopathy was unclear.

**Fig. 1:** Clinicopathological findings. **a**. Skin lesions before treatment. These 1–5-cm erythematous lesions were scattered on the trunk. Lesions larger than the size of a walnut were ulcerated and crusty. Palmer and planter lesions were also present. **b**. Nodular infiltration of the cells from the epidermis to the upper subcutaneous. **c**. Epidermotropism of atypical lymphoid cells. **d**. In the dermis, there is severe inflammation around the venules. Atypical lymphocytes, multinucleated leukocytes, and epithelioid histiocytes are present, but sparse plasma cells. **e**. Immunohistochemical staining for CD8. Lymphocytes were exclusively immunoreactive for CD8. Atypical lymphocytes with nuclear twisting and indentation are also present (*arrows*). **f**. In the bone marrow clot, a number of CD8+ lymphocytes are infiltrating, as indicated by immunohistochemistry. **g**. Atypical lymphocytes and small lymphocytes are seen in the bone marrow smear, suggestive of non-neoplastic cells (*arrowheads*). **h**. *Treponema pallidum* is mainly distributed in the dermis, especially in the perivascular space with histiocytes. Immunohistochemical staining for *Treponema pallidum*

He had the following characteristics at admission: height, 171 cm; weight, 49 kg; blood pressure, 98/63 mmHg; pulse, 90 beats/min; and body temperature, 38.0 °C. His blood examination showed RPR positivity, antibody 5.4 R.U, card method × 4, and *Treponema pallidum* (TP) antigen × 2713.6 U. Anticardiolipin and antinuclear antibody tests were negative. The following results were also obtained: white blood cells, 7470/μL (neutrophils, 83.0 %; lymphocytes, 6.5 %; monocytes, 3.0 %; eosinophils, 3.5 %; basophils, 0.5 %; atypical lymphocytes, 2.5 %; abnormal lymphocytes, 0.0 %; toxic granule +; and hypersegmentation +); red blood cells, 354 × 10^4^/μL; hemoglobin, 10.4 g/dL; hematocrit, 31.7 %; mean corpuscular hemoglobin concentration, 32.8 %; mean corpuscular hemoglobin, 29.4 pg; mean corpuscular volume, 89.5 fL; prothrombin time, 13.8 s, 78 %; prothrombin time-international normalized ratio, 1.12; activated partial thromboplastin time, 41.3 s; fibrinogen, 439 mg/dL; gamma-glutamyl transpeptidase, 80 U/L; lactate dehydrogenase, 180 U/L; total cholesterol, 22 mg/dL; TP, 6.9 g/dL; immunoglobulin (Ig) G, 1879 mg/dL; IgA, 264 mg/dL; IgM, 186 mg/dL; blood urea nitrogen, 8 mg/dL; creatinine, 0.63 mg/dL; C-reactive protein, 5.99 mg/dL; and soluble IL-2 receptor (sIL2R), 1585 U/mL.

The article "Human immunodeficiency virus-positive secondary syphilis mimicking cutaneous T-cell lymphoma" was published in 2015. Journal: Diagn Pathol.

Based on skin biopsy, peripheral T-cell lymphoma not otherwise specified (PTCL-NOS) was suspected (see histological findings). For this pathological diagnosis, sulfamethoxazole-trimethoprim, itraconazole, and prednisolone were prescribed. At admission, syphilis and HIV co-infection was detected on the basis of positivity for the HIV antibody, HIV-RNA of 1.1 × 10^5^ copies/mL, and CD4+ T-cell count of 110/μL. Because he was considered a high-risk AIDS patient, ART consisting of emtricitabine/tenofovir disoproxil fumarate plus efavirenz and methyl prednisolone was initiated. Electron beam irradiation and narrowband ultraviolet B therapy were also performed. Despite partial remission of the skin lesions fever following the therapy, high fever recurred 1.5 months later, and the eruptions had generally spread, producing large amounts of exudate. Persistent fever due to indwelling catheter infection was suspected, for which cefepime to amoxicillin treatment was initiated. The fever reduced significantly, and the eruptions started to disappear. He was discharged from the hospital without undergoing chemotherapy. During the 1-year follow-up at the clinic, he did not experience any symptoms.

### Histological findings

On skin biopsy, diffuse infiltration of atypical lymphoid cells was observed mainly in the upper to mid dermis (Fig. 1b). Some epidermotropism of the atypical lymphoid cells was present (Fig. 1c). The atypical lymphocytes were denser around the skin appendages, and the dermal vessels showed venulitis with extravasation of red blood cells. There were abundant neutrophils, histiocytes, a small number of plasma cells, and eosinophils (Fig. 1d). Nuclear dust was not prominent. Atypical lymphoid cells showed positive immunohistochemical staining for CD3, 1CD7, CD8 (Fig. 1e), granzyme B, and perforin. The Ki-67 labeling index was high. Epstein-Barr virus-encoded RNA was positive only in a few cells. Immunoreactivity for CD4, CD20, CD30, and CD56 were negative.

The article "Human immunodeficiency virus-positive secondary syphilis mimicking cutaneous T-cell lymphoma" was published in 2015. Journal: Diagn Pathol.

In the 4^th^ edition of the WHO classification for tumors, the differential diagnoses in skin lesions with HIV-positive, CD8+ CD30-T-cell proliferation are as follows: primary cutaneous peripheral T-cell lymphoma (primary cutaneous gamma delta T-cell lymphoma or primary cutaneous CD8-positive aggressive epidermotropic T-cell lymphoma), subcutaneous panniculitis-like T-cell lymphoma, mycosis fungoides (rare CD8 subtype), lymphomatoid papulosis (rare CD8 subtype), and lymphoma associated with HIV infection (rare manifestation). The present lesion lacked T-cell receptor (TCR) rearrangement, massive epidermotropism, and panniculitis. Therefore, we initially misdiagnosed the patient with cutaneous PTCL-NOS with a cytotoxic phenotype.

For staging, CD8+ atypical lymphoid cell infiltration (Fig. 1f) and sparse CD4+ cells in the bone marrow clot suggested involvement of CD8+ T-cell lymphoma. Although very few abnormal lymphocytes were present in the bone marrow smear (Fig. 1g), up to 10 % of all nuclear cells were classified as *atypical* lymphocytes, which we assumed to be a reactive change. Therefore, re-evaluation of the skin lesions was performed. The TCR rearrangement of both Jγ and CTβ was polyclonal. The immunohistochemical staining for *Treponema* was re-examined, using the same formalin-fixed paraffin block. Infiltration of numerous spirochetes predominantly in the dermis was observed (Fig. 1h). On the basis of these data and the clinical course, we finally concluded that the skin lesions were not neoplastic and were secondary syphilids that mimicked T-cell lymphoma in an HIV-positive host.

### Discussion

Ordinary secondary syphilis presents various skin manifestations. However, approximately 80 % of patients show superficial lichenoid/psoriasiform inflammation with a plasma cell-, lymphocyte-, and histiocyte-dominant pattern. *Treponema pallidum* distribution is also epitheliotropic [18]. In contrast, inflammatory cells are deeper and more complicated in malignant secondary syphilis. Lues maligna is the more common name for malignant secondary syphilis in dermatology and is characterized by dermal plasma cells admixed with lymphocytes, histiocytes, and neutrophils—neutrophilic venulitis is described as a pattern of lues maligna—but spirochetes are infrequently found [19, 20]. An appropriate *Treponema* immunohistochemical staining technique might be needed for diagnosis.

The article "Human immunodeficiency virus-positive secondary syphilis mimicking cutaneous T-cell lymphoma" was published in 2015. Journal: Diagn Pathol.

In our case, ART was not effective but a combination of ART and antibiotics such as penicillin-G improved the symptoms, while RPR antibody 5.4 R.U tested negative. Venereal Disease Research Laboratory/Rapid Plasma Reagin (VDRL/RPR) titers have been reported to range between 1:16 and 1:4096 in HIV-negative classical malignant syphilis [3]. In any event, an HIV-positive patient’s sample requires diluted re-examination for prozone phenomenon. RPR was originally designed as a method for detecting autoantibodies, and its titer reflects tissue inflammation level caused by *Treponema pallidum* infection. Therefore, in HIV-positive cases, immunodeficiency may lead to low titer-positive and prolonged negative conversion. We also think that systemic CD4+ lymphocytopenia caused by a severe HIV infection and some hypercytokinemia caused by lues maligna might play a significant role on the appearance of numerous CD8+ atypical lymphocytes and fewer plasma cells (Table 1).

**Table 1:** Number of CD4+ cells, results of the rapid plasma reagin (RPR) test for *Treponema pallidum*, and human immunodeficiency virus RNA

*PSL* prednisolone, *EB* electron beam, *UV* narrowband ultraviolet B, *AMPC* amoxicillin, *CFPM* cefepime, *ART* antiretroviral therapy, *TDF/FTC+EFV* emtricitabine/tenofovir disoproxil fumarate plus efavirenz, *ND* not done, *RPR* rapid plasma reagin, *HIV* human immunodeficiency virus

## Conclusions

When ulcerated skin lesions are observed in a patient with syphilis and HIV co-infection, a diagnosis of lues maligna should be considered before diagnosing the patient with cutaneous lymphoma, even if there is an abundance of CD8+ lymphocytes without plasma cells. Slight neutrophilic venulitis might be an important finding. The diagnosis could be confirmed by the serological syphilis test (STS) or *Treponema pallidum* hemagglutination (TPHA) test (both positive), immunohistochemical positivity for *Treponema pallidum*, and TCR polyclonality in the skin lesion. Cases of co-infections with malignant syphilis and HIV have been on the rise, and delayed diagnosis is dangerous not only for the patient but also for public health. The present case demonstrates that pathologists should be aware of the possibility of lues maligna with HIV, mimicking cutaneous T-cell lymphoma.

The article "Human immunodeficiency virus-positive secondary syphilis mimicking cutaneous T-cell lymphoma" was published in 2015. Journal: Diagn Pathol.

## Consent

Written informed consent was obtained from the patient for publication of this Case Report and any accompanying images. A copy of the written consent is available for review by the Editor-in-Chief of this journal. Our hospital Ethics Committee provided ethical approval for the publication of this report.

## Abbreviations

ART: Antiretroviral therapy
HIV: Human immunodeficiency virus
Ig: Immunoglobulin
PTCL-NOS: Peripheral T-cell lymphoma not otherwise specified
RPR: Rapid plasma reagin
STS: Serological syphilis test
sIL2R: Soluble IL-2 receptor
TCR: T-cell receptor
TP: *Treponema pallidum*
TPHA: *Treponema pallidum* hemagglutination
VDRL/RPR: Venereal Disease Research Laboratory/Rapid Plasma Reagin
WHO: World Health Organization

## References

[1] Fisher DA, Chang LW, Tuffanelli DL (1969). Lues maligna. Presentation of a case and a review of the literature. Arch Dermatol.

[2] Lejman K, Starzycki Z (1972). Syphilis maligna praecox. A case report. Br J Vener Dis.

[3] Kumar B, Muralidhar S (1998). Malignant syphilis: a review. AIDS Patient Care STDS..

[4] Sands M, Markus A (1995). Lues maligna, or ulceronodular syphilis, in a man infected with human immunodeficiency virus: case report and review. Clin Infect Dis..

[5] Zetola NM, Engelman J, Jensen TP, Klausner JD (2007). Syphilis in the United States: an update for clinicians with an emphasis on HIV coinfection. Mayo Clin Proc.

[6] Osato K, Nagao T, Inuzumi K, Araki H, Kawai K (2001). Recent trend of syphilis infection in HIV-1 infected patients. Japanese Journal of Sexually Transmitted Diseases..

[7] Pialoux G, Vimont S, Moulignier A, Buteux M, Abraham B, Bonnard P (2008). Effect of HIV infection on the course of syphilis. AIDS Rev..

[8] Buchacz K, Patel P, Taylor M, Kerndt PR, Byers RH, Holmberg SD (2004). Syphilis increases HIV viral load and decreases CD4 cell counts in HIV-infected patients with new syphilis infections. AIDS..

[9] Jurado RL, Campbell J, Martin PD (1993). Prozone phenomenon in secondary syphilis. Has its time arrived?. Arch Intern Med.

[10] Lynn WA, Lightman S (2004). Syphilis and HIV: a dangerous combination. Lancet Infect Dis..

[11] Hodak E, David M, Rothem A, Bialowance M, Sandbank M (1987). Nodular secondary syphilis mimicking cutaneous lymphoreticular process. J Am Acad Dermatol..

[12] Park SY, Kang JH, Roh JH, Huh HJ, Yeo JS (2013). Kim do Y. Secondary syphilis presenting as a generalized lymphadenopathy: clinical mimicry of malignant lymphoma. Sex Transm Dis.

[13] Egbers RG, Do TT, Su L, Helfrich YR, Gudjonsson JE (2011). Rapid clinical change in lesions of atypical cutaneous lymphoproliferative disorder in an HIV patient: a case report and review of the literature. Dermatol Online J..

The article "Human immunodeficiency virus-positive secondary syphilis mimicking cutaneous T-cell lymphoma" was published in 2015. Journal: Diagn Pathol.

[14] Schartz NE, De La Blanchardiére A, Alaoui S, Morel P, Sigaux F, Vignon-Pennamen MD (2003). Regression of CD8+ pseudolymphoma after HIV antiviral triple therapy. J Am Acad Dermatol..

[15] Tosca A, Stavropoulos PG, Hatziolou E, Arvanitis A, Stavrianeas N, Hatzivassiliou M (1990). Malignant syphilis in HIV-infected patients. Int J Dermatol..

[16] Muche JM, Toppe E, Sterry W, Haas N (2004). Palpable arciform migratory erythema in an HIV patient, a CD8+ pseudolymphoma. J Cutan Pathol..

[17] Swerdlow SH, Campo E, Harris NL, Jaffe ES, Pileri SA, Stein H, et al. WHO classification of tumours of haematopoietic and lymphoid tissues. 4th ed. World Health Organization. Lyon, France: IARC Press; 2008.

[18] Martín-Ezquerra G, Fernandez-Casado A, Barco D, Jucglà A, Juanpere-Rodero N, Manresa JM (2009). *Treponema pallidum* distribution patterns in mucocutaneous lesions of primary and secondary syphilis: an immunohistochemical and ultrastructural study. Hum Pathol..

[19] Don PC, Rubenstein R, Christie S (1995). Malignant syphilis (lues maligna) and concurrent infection with HIV. Int J Dermatol..

[20] Yanagisawa N, Ando M, Imamura A, Akagi K, Horiguchi S, Suganuma A (2011). Pathologically confirmed malignant syphilis in an HIV-infected patient. Intern Med..

